The article "The Intervention of Music Therapy on Behavioral Training of High-Functioning Autistic Children under Intelligent Health Monitoring" was retracted in 2023. Reasons: signs of a paper mill; suspected computer-generated content; unreliable results or conclusions; lack of ethics approval or compliance.

# The Intervention of Music Therapy on Behavioral Training of High-Functioning Autistic Children under Intelligent Health Monitoring

**DOI:** 10.1155/2022/5766617

**Published:** 2022-05-13

**Authors:** Rugui He

**Affiliations:** College of Music, Guizhou Normal University, Guiyang, 551700 Guizhou, China

## Abstract

Autism is a serious and widespread developmental disorder in children. With the increase of autistic children every year, it is necessary to study a set of effective music therapy activities that can penetrate into life to help autistic children's rehabilitation training. This paper aims to study the behavioral training of high-functioning autistic children with music therapy intervention under intelligent health monitoring. The autistic children were selected and divided into experimental group and control group. According to the psychological and physiological characteristics of five autistic children aged 5-7 years in the experimental group, the music therapy activity plan was designed, and the experimental intervention was carried out by combining individual music therapy and group music therapy. Compared with the control group, this paper explores the effect of music on the treatment of children with autism. The experimental results of this paper show that the language, social, cognitive, and behavioral problems of autistic children under music therapy under intelligent health monitoring have been significantly improved, and their emotional response ability has improved the most, increasing by 34%. Communication ability was next, increased by 20.3%; motor coordination ability increased by 20%; and cognitive ability improved by 11%. It can be explained that the four aspects of language, social interaction, cognition, and behavior have been significantly improved after music therapy.

## 1. Introduction

Due to the pollution of various ecological environments, the environment in which people live is getting worse and worse, and the probability of pregnant women being diagnosed with deformed children during pregnancy is also greatly increased. The number of births of children with congenital disabilities is as high as 800,000 to 1.2 million each year, accounting for 4% to 6% of the country's total population. Especially in children with Down syndrome, the annual cost of treatment alone exceeds 2 billion yuan. This is not only a disaster for a family, but also a burden to society. Children with Down syndrome are often accompanied by certain behavioral disorders, such as hyperactive behavior, fearful behavior, autistic behavior, obsessive-compulsive behavior, and aggressive behavior. These behaviors have caused them serious adaptation disorders, so they need to be corrected and helped by certain means. And using music as a means of therapy is more loved and accepted by children in a more relaxed and cheerful environment. Intelligent health monitoring provides more objective and precise experimental data for the study of music therapy intervention on behavioral training of high-functioning autistic children [1].

Because high-functioning autistic children are a disease caused by chromosomal abnormalities, drug treatment has a little effect [2]. Therefore, while music therapy can replace the effect of drugs to a certain extent, effective music therapy methods can also help children to produce therapeutic effects without side effects. As a new discipline, music therapy still lacks a solid theoretical foundation and clinical practice experience in the field of children with special disabilities. Therefore, the application of music therapy to the clinical practice of high-functioning autistic children, especially the rehabilitation training of children's behavioral disorders, is of great significance for the development of music therapy in the field of high-functioning autistic children and obtaining valuable clinical experience.

The innovation and value of this paper are mainly reflected in the following two aspects. First, this paper discusses the related issues of music therapy's intervention on mentally handicapped children's emotional disorders by means of empirical research, the technical methods and characteristics of music therapy for mentally handicapped children, and the effect of music therapy on mentally handicapped children's emotional intervention and matters needing attention. It provides theoretical data for the research and application of Chinese music therapy in the education of children with intellectual disabilities. Secondly, domestically, behavior modification, medical rehabilitation, and other methods are mainly used for mentally handicapped children. These methods can correct the bad behavior of intellectually handicapped children, but it is difficult to substantially improve their psychological and emotional problems. This study starts with the emotional factors that affect mentally handicapped children's psychology and behavior and promotes their physical and mental development and social adaptation by improving their emotional expression and self-management abilities. Therefore, it provides a more operable and practical practice program for the education and training of mentally handicapped children.

## 2. Related Work

People with autism spectrum disorder (ASD) produce impoverished personal narratives. Allyssa developed an intervention to improve parental conversations with sons/daughters with ASD to improve children's narratives [3]. Because the core symptom of ASD is social communication and communication impairment, the behavior and interests are stereotyped and narrowed, but there is no significant change in this symptom. Nonpharmacological interventions appear to benefit many patients without the side effects usually associated with drugs. Music-based experiences may benefit intensive care patients. Golino A J examines the effect of an active music therapy intervention on physiological parameters and self-reported pain and anxiety levels in intensive care unit patients [4]. Although his music therapy interventions have been greatly improved in intensive care unit patients, individual differences among study subjects have not been thoroughly studied. The Storch study found that 1 in 63 children/teens had an autism spectrum disorder (ASD). It is characterized by impaired cognition, communication, and/or social responsiveness and interaction. He has developed and researched a number of interventions to target social skills in children and adolescents with ASD [5]. The Sadeghi S study aimed to assess the impact of a home-based remote intervention SPARK program on improving motor performance and reducing the severity of autism symptoms in children with high-functioning ASD. The study adopted a quasi-experimental pretest and posttest design without a control group [6]. While his SPARK program improved motor skills in children with ASD, it did little to reduce the severity of autism symptoms. Music plays an important role in everyone's life, and the Barnes study found that some health-care providers may dislike music therapy and its positive benefits to the environment, patients, caregivers, and health-care providers [7]. However, his integrative music therapy (IMT) has been shown to be effective in a variety of settings, but provides little treatment for behavioral, emotional, physical, psychological, and psychosocial needs. Music therapy is a separate discipline within the interdisciplinary field of science and art. Katui A's research demonstrates the theoretical underpinnings of music therapy in the fields of human psychology and music pedagogy, and the development of music therapy models derived from these theoretical approaches. Improvisation in these models plays a key role in skill acquisition and improvement [8]. Music therapy abandons the traditional diagnosis mode that only focuses on the pathological changes of the patient, and at the same time heals the patient's body and mind, so as to achieve a better therapeutic effect. The Zaurati M study found that music therapy has analgesic effect and has been clinically applied in the puerperium to divert attention from labor pain during the puerperium [9]. Although studies have found that music therapy is used to relieve tension during pregnancy, the negative emotions that may arise can have adverse effects on the mother and the fetus.

## 3. Music Therapy under Intelligent Health Monitoring

### 3.1. Overall Design Scheme

The system consists of four parts: a wearable detection module for physiological parameters, an intelligent medicine box module for processing and drug management of the main controller, a software monitoring module for a smartphone, and a remote monitoring server module [10–11]. The overall structure of the system is shown in Figure 1.

The physiological parameter acquisition module includes four detection sensors: pulse sensor, blood pressure sensor, heart rate sensor, and temperature sensor [12]. The pulse sensor is the SC0073B pulse sensor used. The blood pressure sensor uses a resistive MPS3117-006GA, and the heart rate sensor uses a finger heart rate sensor HRM-2511E.The smartphone software monitoring module includes a user information management module, a physiological data processing module, a drug management module, and an abnormal data alarm module [13]. The remote monitoring server module, as the PC side, deploys the designed web page on the Tomcat server on the PC side, and the remote medical staff can use the computer browser to obtain the public network IP to observe the physiological condition of the ward.

### 3.2. Algorithms Related to Intelligent Health Monitoring

#### 3.2.1. Effective Independence Law

The effective independence method (EFI) targets the linearly independent contribution of each sensor point to the modal vector. It optimizes the Fisher information matrix to keep the modal vector of interest as linearly independent as possible with the fewest measurement points, so as to obtain the maximum modal information with limited sensors [14–15].

Assuming that each modal vector in the modal matrix of the theoretical model is independent and orthogonal, the output of the initial selection of *s* candidate measurement points is

(1) $$\begin{array}{c} U_{s}=\varphi_{s}q. \end{array}$$

The modal coordinates are estimated as

(2) $$\begin{array}{c} \hat{q}={\left[\varphi_{s}^{T}\varphi_{s}\right]}^{-1}\varphi_{s}u_{s}. \end{array}$$

where *u*_*s*_ is the output of the initial selection of candidate measuring points; *φ*_*s*_ is the part of the modal matrix *φ* on the candidate measuring points; and $\hat{q}$ is the modal coordinate vector [16].

If the actual number of measuring points selected is *m* (*m* < *s*), then, the problem can be expressed as how to find *m* measuring points from *s* selectable measuring points. And the modal linear independence measured at these *m* points is the best estimate of the modal space [17]. Here, the covariance of the errors is taken as the best estimate. Taking into account the effect of noise, the output formula is rewritten as

(3) $$\begin{array}{c} u_{s}=\varphi_{s}q+N. \end{array}$$

Then, the covariance of the estimated error is

(4) $$\begin{array}{c} P=E\left[\left(q-\hat{q}\right){\left(q-\overset{\wedge }{q}\right)}^{T}\right]=\varphi_{s}^{T}\left(\varphi_{0}\varphi_{s}\right)=Q^{-1}, \end{array}$$

where *Q* is the Fisher information matrix. Assuming that the noise is Gaussian white noise, then

(5) $$\begin{array}{c} Q=\frac{\varphi_{s}^{T}\varphi_{s}}{\varphi_{0}^{2}}=\frac{A}{\varphi_{0}^{2}}. \end{array}$$

It can be seen from Formula (5) that the minimum value of the covariance *P* of the estimation error is equivalent to the maximum value of the Fisher information matrix *Q*. That is, the trace (trace) of matrix *A* in Formula (6) or the estimation when its determinant value is the largest is an unbiased estimation [18].

Matrix *A* can be written as

(6) $$\begin{array}{c} A=\overset{s}{\underset{i=1}{\sum }}{\left[\varphi_{s}^{i}\right]}^{T}\left[\varphi_{s}^{i}\right]=\overset{s}{\underset{i=1}{\sum }}A^{i}\;, \end{array}$$

where *A*^*i*^ represents the contribution of the *i*-th degree of freedom to matrix *A*.

The characteristic formula of the solution matrix *A* is

(7) $$\begin{array}{c} \left(\text{A}-\lambda I\right)\varphi =0, \end{array}$$

(8) $$\begin{array}{c} \varphi^{T}A\varphi =\lambda ,\varphi^{T}\varphi =I\;, \end{array}$$

(9) $$\begin{array}{c} \varphi^{T}\lambda \varphi =A^{-1}. \end{array}$$

Construct matrix *E*:

(10) $$\begin{array}{c} E=\varphi_{s}\varphi \lambda^{-1}{\left(\varphi_{s}\varphi \right)}^{T}=\varphi_{s}A^{-1}\varphi_{s}^{T}, \end{array}$$

(11) $$\begin{array}{c} E=\varphi_{s}{\left(\varphi_{s}^{T}\varphi \right)}^{-1}\varphi_{s}^{T}. \end{array}$$

Obviously, in Formula (11), *E*^2^ = *E* and *E* are idempotent matrices whose eigenvalues are 1 or 0, and the trace is equal to rank; that is, tr(*A*) = rank(*A*). The *i*-th element on its diagonal represents the contribution of the *i*-th degree of freedom or measurement point to the rank of matrix *φ*_*s*_, that is, the contribution to matrix *A* [19]. Write the diagonal elements of *E* as a column vector as

(12) $$\begin{array}{c} EI={\left[E_{11}\;E_{22},\cdots ,E_{ss}\right]}^{T}. \end{array}$$

Among them, the size of each element represents the relative size of the contribution of each degree of freedom or measurement point to the rank in the matrix.

#### 3.2.2. QR Decomposition Method

It can be known from the effective independence method that when the Fisher information matrix *Q* takes a maximum value, the covariance *P* of the estimation error is extremely small.

Here, the 2-norm ‖*Q*‖_2_ is selected as

(13) $$\begin{array}{c} {\left\|Q\right\|}_{2}={\left\|\varphi_{s}^{T}\varphi \right\|}_{2}. \end{array}$$

By meeting the requirement of *Q*, according to the relevant matrix theory, the column pivot QR decomposition is a simple and effective method when selecting a matrix column vector group with the largest norm subset [20–21].

Assuming that the subset of measurable degrees of freedom of the mode shape matrix obtained by the finite element model is medium, *φ*∈*R*^*n*∗*n*^, and *r*(*φ*) = *m*, the matrix column *φ* is full rank [22]. Perform column pivot QR decomposition on *φ*^*T*^, and select a subset of column vector groups as

(14) $$\begin{array}{c} \varphi^{T}E=\text{QR}=\left[\begin{array}{cc} R_{11} & R_{1n}\\ 0 & R_{mm} \end{array}\right], \end{array}$$

where *E* is the permutation matrix, *E∈R*^*n*∗*n*^, *Q∈R*^*m*∗*n*^, *R∈R*^*m*∗*m*^. The first *m* columns of matrix AA correspond to a set of row vectors with larger norm in matrix BB. The *m* measurable degrees of freedom are a set of measurable degrees of freedom that make the Fisher information matrix have a larger norm [23].

#### 3.2.3. Modal Kinetic Energy Method

The modal kinetic energy method (MKE) configures the sensor by comparing the modal kinetic energy among the test degrees of freedom and selecting the degree of freedom with the larger modal kinetic energy. In this way, the signal-to-noise ratio of the structural dynamic response signal test can be improved [24–25]. Assuming a mode matrix with *l*-order mode shape, the modal kinetic energy corresponding to the *k*-th mode of the *i*-th test degree of freedom is defined as

(15) $$\begin{array}{c} \text{MK}{\text{E}}_{\text{ik}}=\varphi_{ik}\overset{\text{i}}{\underset{\text{j}=1}{\sum }}{\text{M}}_{\text{ij}}\varphi_{jk}\;, \end{array}$$

where *φ*_*ik*_ and *φ*_*jk*_ are the components of the *k*-th mode in the *i*-th test degree of freedom and the *k*-th mode in the *j*-th test degree of freedom [26] and *M*_*ij*_ is the corresponding element in the mass matrix. The modal kinetic energy *MKE*_*dof*_ of each test degree of freedom is

(16) $$\begin{array}{c} {\text{MKE}}_{\text{dof}}=\mathrm{diag}\left(\varphi_{s}\varphi_{s}^{T}\text{M}\right). \end{array}$$

According to the modal kinetic energy of the obtained optional degrees of freedom, the final configuration point of the sensor can be determined by selecting the m maximum test points in the modal kinetic energy [27–28].

#### 3.2.4. Modal Strain Energy Method

In order to facilitate parameter identification, the basic principle of the modal strain energy method (MSE) states that the sensor should be configured on the degrees of freedom with large modal strain energy in the structure [29–30]. For a dynamic structure with *n* degrees of freedom, the strain energy matrix *E* = (*E*_*ij*_)_*n*∗*n*_ for each degree of freedom on the structure is defined as

(17) $$\begin{array}{c} E=\frac{1}{2}u^{T}Ku=\frac{1}{2}{\left(\varphi q\right)}^{T}K\varphi q=\frac{1}{2}q^{T}\varphi^{T}K\varphi q, \end{array}$$

where *φ* is the normalized mode shape matrix; *u* is the displacement matrix; *q* is the normalized coordinate matrix; and *K* is the stiffness matrix.

Modal strain matrix *E*_MSE_ = *φ*^T^K*φ* is defined as

(18) $$\begin{array}{c} E_{MSE}=\left[\begin{array}{ccc} \underset{i,j}{\sum }\varphi_{i1}k_{ij}\varphi_{j1} & \underset{i,j}{\sum }\varphi_{i1}k_{ij}\varphi_{j2} & \underset{i,j}{\sum }\varphi_{i1}k_{ij}\varphi_{jn}\\ \underset{i,j}{\sum }\varphi_{i2}k_{ij}\varphi_{j1} & \underset{i,j}{\sum }\varphi_{i2}k_{ij}\varphi_{j23} & \underset{i,j}{\sum }\varphi_{i2}k_{ij}\varphi_{jn}\\ \underset{i,j}{\sum }\varphi_{\text{in}}k_{ij}\varphi_{j1} & \underset{i,j}{\sum }\varphi_{\text{in}}k_{ij}\varphi_{j1} & \underset{i,j}{\sum }\varphi_{\text{in}}k_{ij}\varphi_{j1} \end{array}\right], \end{array}$$

where *k*_*ij*_ is the stiffness coefficient between node *i* and node *j*; *φ*_*ij*_ is the component of the *j*-th order matrix on the *i*-th degree of freedom; and the matrix *E*_*MSE*_ is a symmetric matrix. The *i*-th row and *j*-column elements in the matrix represent the strain energies associated with the *i*-th and *j*-order modes. The sum of all elements in the *i*-th row represents the total modal strain energy associated with the *i*-th mode. Select *m* from the *n* degrees of freedom possessed by the dynamic structure, and use the set of *m* measuring points with the largest modal kinetic energy as the sensor configuration point.

#### 3.2.5. Guyan Model Reduction Method

The Guyan model reduction method divides the degrees of freedom of the model, including the main degree of freedom and the secondary degree of freedom, in which the influence of the quality of the secondary degree of freedom on the structure is ignored. The expression for modal reduction is

(19) $$\begin{array}{c} \left[\begin{array}{cc} k_{t} & k_{t0}\\ k_{0t} & k_{0} \end{array}\right]\left[\begin{array}{c} \varphi_{t}\\ \varphi_{0} \end{array}\right]=\omega^{2}\left[\begin{array}{cc} m_{t} & 0\\ 0 & 0 \end{array}\right]\left[\begin{array}{c} \varphi_{t}\\ \varphi_{0} \end{array}\right], \end{array}$$

where *φ*_*t*_ is the mode matrix corresponding to the main degree of freedom; *k*_*t*_ is the stiffness matrix corresponding to the main degree of freedom; and *m*_*t*_ is the mass matrix corresponding to the main degree of freedom.

By reducing, we get

(20) $$\begin{array}{c} {\text{k}}_{\text{t}}\varphi_{t}=\omega^{2}m_{t}\varphi_{t}. \end{array}$$

Among them, *k*_*t*_ = *k*_*t*_ − *k*_*t*0_*k*_*t*0_^−1^*k*_0*t*_. Assuming that *m* test points are selected as the sensing configuration points, the measurement point group corresponding to the main degree of freedom is (*t*_1_, *t*_2_, ⋯, *t*_*m*_).

## 4. Behavioral Intervention Experiment of Music Therapy on High-Functioning Autistic Children

### 4.1. Research Questions

Restricted by their own defects, mentally handicapped children have many difficulties in social and school adaptation, resulting in more emotional problems. On the other hand, because intellectually handicapped children cannot make corresponding emotional responses to external stimuli, they are prone to negative emotions such as anxiety and depression, which in turn affect the interpersonal communication, learning, and life of intellectually handicapped children. Almost all studies have shown that children with intellectual disabilities have higher levels of anxiety, depression, and loneliness than ordinary children. About 10%-60% of children with intellectual disabilities have generalized anxiety disorder. They are prone to nervousness, anxiety, depression, irritability, lack of concentration, low self-focus, and feeling fatigued. For the treatment of emotional problems in children with intellectual disabilities, sensory integration training, behavior modification, and other treatment methods are usually used in educational practice. These methods can correct the bad behaviors of children with intellectual disabilities, but their effect is still very limited in improving the emotional function and emotional expression of children with intellectual disabilities. Because of its unique effect on emotions, music therapy can bypass language constraints and act on mentally and psychologically of mentally handicapped children. Its negative emotions can be adjusted and improved, and positive emotions and emotional literacy can be obtained, and its psychology and behavior can also be reasonably improved.

In this study, five mentally handicapped children with emotional disorders were used as the subjects. According to the principles and methods of developmental psychology and art therapy, music therapy experiments aimed at improving emotional disorders were carried out on these subjects. The purpose of music therapy is to improve autistic children's cognition, improve mood and eliminate symptoms (physical, psychological, behavioral, expression, and communication barriers), and improve their self-awareness and life adaptability.

### 4.2. Research Objects

The object of this experiment is to select five mentally handicapped children with typical emotional disorders from a mentally handicapped school in Jinan. The choice of the form of music therapy is based on the problem or disorder of the autistic child, using individual lessons, group lessons, group lessons, or alternating individual lessons and group lessons. They were all under the age of 18, and their typical emotional and behavioral manifestations were as follows:

Xiao Y, female, 13 years old, has moderate intellectual disability, difficulty in language expression, timidity, sensitive anxiety, irritability, emotional instability, self-injury behavior, and poor physical coordination

Little F, female, 15 years old, with mild intellectual disability, emotional irritability, self-injury, and aggressive behavior

Little M, male, 16 years old, moderate intellectual disability, language disorder, emotional disorder, fearful and nervous about unfamiliar environment, anxious, shy and introverted, emotionally unstable, easy to lose temper, and depression

ZY, male, 14 years old, mild mental retardation, language difficulties, easy to lose his temper when emotionally unstable, covering his ears for a long time “humming”, and stereotyped movements

Xiao W, male, 12 years old, with severe intellectual disability, language disorder, emotional anxiety and tension, self-injury and aggressive behavior, hyperactivity, and stereotyped movements.

Method for testing the effectiveness of music therapy teaching: The effectiveness of music therapy is to conduct a variety of abilities (inside music and abilities outside music) and individual tests for individual autistic children, such as music abilities, language, cognition, and communication or the ability to communicate. Due to illnesses and travel, the number of treatments ZY and Xiao W received did not reach 20 times, and their treatment data could not be investigated quantitatively, but were only used for qualitative analysis. The focus of this study is to explore the effects of music on the treatment of children with autism through experimental research on music therapy for children with autism.

### 4.3. Staged Treatment Arrangements

This study used a combination of individual music therapy and group music therapy, the childhood autism rating scale (CARS) and the autism treatment evaluation scale (ATEC). Taking into account the CARS score and ATEC score of the children, combined with the interview records of parents and teachers, and the characteristics of behavioral disorders observed by the researchers, this paper also refers to the existing relevant research. For individual music therapy and group music therapy, this paper has targeted arrangements for music therapy activities. The goals of music therapy for children with autism also need to be set as far as possible in line with the educational goals of other disciplines in special education schools. The problems that children with autism need to solve in other courses are integrated into music therapy to solve together, which is the essential need for music therapy to take root in special education schools.

#### 4.3.1. Individual Music Therapy

Individual music therapy is about establishing a one-on-one therapeutic relationship. In individual music therapy, the relationship between the therapist and the patient is critical and often determines the success or failure of therapy. The structure of music therapy practice for children with autism is shown in Figure 2.

It can be seen from Figure 2 that the relationship between the therapist and the autistic child should be based on empathy, understanding, trust, and support and music is the link between the therapist and the autistic child.

#### 4.3.2. Group Music Therapy

Group music therapy is mainly to let children with autism understand the concept of cooperation. Through music therapy activities, children can learn to communicate with others, share, obey order, and learn positive behaviors such as correct manners. During this process, autistic children need to be accompanied by their parents to assist the therapist in their work and help the group complete various instructions from the therapist. But it cannot be replaced. The therapist and the autistic child should have an equal and cooperative relationship, actively participate in the treatment process, and help the child achieve the purpose of treatment. The seating arrangement should form a circle so that every member, including the therapist, has an equal position. A schematic diagram of the dynamic relationship of the group therapy group is shown in Figure 3.

It can be seen from Figure 3 that the evaluation scheme of music therapy for children with intellectual disabilities in this experiment was formulated. According to the international general children's music therapy procedures, the whole process of tracking and recording of each child was carried out, and the single-subject experimental method of before and after control was adopted for research and evaluation. Fill out the daily schedule form and detailed records after each treatment. The date, time, and record must be filled in the daily schedule to analyze the whole process of treatment. The inductive analysis of the data needs to consider two levels:

1. Target behavior duration: Calculate the duration of each target behavior in minutes
2. Frequency of target behaviors: The number and time of occurrences of the same target behavior are arranged together. The records of the whole process of each subject's treatment experiment are bound into a table, and the independent variables in the table are the intervention methods of the music therapist to the positive reinforcement music training of the experimental subjects. The dependent variable is the change of the subject's musical performance ability and behavioral performance ability after the music experience

### 4.4. Research Results

#### 4.4.1. Experimental Results and Data Analysis and Processing

Significance testing was performed using the signed-rank sum test in nonparametric tests. The Wilcoxon test has no requirements on the form of the data distribution and can be considered when the data does not meet the normal distribution requirements of the *t* test. Only 5 children were selected in the experimental group. Statistically, the sample size was too small, so the signed-rank sum test method of nonparametric test was selected, which may weaken the interpretation of the data.

*(1) Comparison of Total ATEC Scores Before and After the Experiment*. The ATEC scores before and after the ATEC test of the experimental group and the control group were drawn into a visual map for comparative analysis.  Figure 4 shows the comparison of the total ATEC score before and after the experiment.

As shown in Figure 4, the 5 children in the experimental group all improve to varying degrees, while the children in the control group did not improve at all. Among them, the improvement of SY2, SY3, and SY4 in the experimental group was more obvious, but the improvement of SY1 and SY5 was not obvious.

*(2) Signed-Rank Sum Test of ATEC Total Scores Before and After the Experiment*. The ATEC total scores of the children in the experimental group and the control group were input into SPSS 17.0 software for signed-rank sum test. The results are shown in Table 1 and Table 2:

From Table 1 and Table 2, it can be seen that there was no significant difference in the total ATEC score of the children in the control group at *p* ≤ 0.05, while there was a significant difference in the pre- and posttest scores of the children in the experimental group (*p* ≤ 0.05).

### 4.5. The Scores of Each Subscale of ATEC Before and After the Experiment

Figures 5 and 6 show the comparison charts of the pretest and posttest scores of each subscale of ATEC between the experimental group and the control group.

As shown in Figures 5 and 6, after a period of music therapy activity experiment, the scores of each subscale of ATEC of the 5 children in the experimental group were improved to varying degrees. Among them, the social subscales of SY2, SY3, and SY4 improved significantly. The improvement of each subscale of SY1 and SY5 was not as obvious as that of SY2, SY3, and SY4. Children in the control group showed little improvement.

### 4.6. Signed-Rank Sum Test Results of Pre- and Posttest Scores for Each Subscale of ATEC

The scores of each subscale of ATEC in the experimental group and the control group before and after the experiment were compared by the signed-rank sum test. The results can be seen from Table 3 and Table 4; the children in the control group did not achieve significant differences in all aspects of the ATEC scale in the pre- and posttest. However, there were significant differences in the scores of the four subscales of language, social interaction, cognition, and behavior in the experimental group.

According to the statistical results of the signed-rank sum test, the language, social, cognitive, and behavioral status of the control group remained at the same level. The children in the experimental group had significant improvements in language, social interaction, cognition, and behavior after music therapy.

### 4.7. Case Study

Through 22 sessions of music therapy training for a total of 2640 minutes, the five tested children have significantly improved their musical ability and mental ability, especially their emotions, communication, and musical sensibility. The specific situation is presented in a case report.  Figure 7, Figure 8, and Figure 9 show the emotional and behavioral performance of Xiao Y, Xiao F, and Xiao M before and after music therapy, respectively.

From the test results, it can be seen that Xiao M's emotional response ability has improved the most, increasing by 34%, followed by communication ability, which has increased by 20.3%, motor coordination ability has increased by 20%, and cognitive ability has improved by 11%. It can be seen that the five subjects experienced great changes in their mood and behavior after six months of music therapy training. In particular, the cognition, expression, and control of emotions have been significantly improved. This experiment proves that music therapy can regulate and improve the negative emotions of children with mild and moderate intellectual disabilities and can promote the development of positive emotions in children with mild and moderate intellectual disabilities. And through the treatment and intervention of these children, the frequency of their bad behaviors has also been reduced to varying degrees, and the interpersonal skills can also be improved to a certain extent. It can be shown that music therapy activities have a certain improvement effect on the problem behaviors of these five cases, so music has a positive impact on the treatment of children with autism.

## 5. Conclusions

Through the analysis of the experimental results, it can be seen that music is helpful for the rehabilitation of children with autism. The beneficial effects of music on the treatment of autism in children are shown in the following aspects. After the signed-rank sum test by SPSS17.0 software, it was found that the language, social, cognitive, and behavioral problems of autistic children have significant improvement. Judging from the quantitative results, it can be seen from the four observation points of the subject's pre- and posttest data receiving music therapy activities, the test data during the experiment, and the language, social interaction, cognition, and behavior of children with autism. Music enables children with autism to use music to communicate in the absence of language. It then gradually introduces language training through other activities of music, such as singing and reciting the rhythm of songs, so as to achieve the improvement or rehabilitation of language communication ability. Judging from qualitative data, music can create a relaxed and pleasant space for activities and make autistic children gradually become confident with the help of music. The physical rhythm of children with autism is induced by the stimulation of music to regulate the movement ability and improve the movement coordination to a certain extent. Children with autism can receive friendly information in a stress-free and pleasant music atmosphere and are driven to learn and communicate. The operability, feasibility, flexibility, and various behavior problems of this paper have been improved to a certain extent, and it has immediate and continuous effects and good stability. Children with autism can relax and accept external stimuli freely and respond in music. It is hoped that this will promote the research and development of the treatment of children with autism, help children with autism to regulate their emotions, develop adaptive behaviors, experience life, learn to be independent, improve their quality of life, and integrate into society as soon as possible. Inspired by music, autistic children externalize their inner emotions and emotions that cannot be expressed in words through behavior. In the later stage, if we can conduct long-term observational research with large samples, collect more relevant information, establish a more complete evaluation mechanism, and do more detailed coding analysis of the obtained experimental results, it is believed that more valuable statistical data can be obtained.

## Figures and Tables

**Figure 1:** Overall architecture diagram of the system.

**Figure 2:** The structure of music therapy practice for children with autism.

**Figure 3:** Schematic diagram of the dynamic relationship of the group therapy group.

**Figure 4:** Visual diagram of the comparison of the total ATEC score before and after the test group and the control group.

**Figure 5:** Visual chart of the scores of each subscale of ATEC before and after the five children in the experimental group.

**Figure 6:** Visual chart of the scores of each subscale of ATEC before and after the 5 children in the control group.

**Figure 7:** The emotional and behavioral performance of Xiao Y's musical performance ability before and after music therapy.

**Figure 8:** The emotional and behavioral performance of Xiao F before and after music therapy.

**Figure 9:** Music expressive ability of Xiao M before and after music therapy, emotional and behavioral expressive ability.

**Table 1:** Sign-rank sum test results of ATEC total scores of children in experimental group.

		*N*	Rank mean	Rank sum	*Z*	Asymptotic significance (bilateral)
ATEC total score posttest —ATEC total score pretest	Negative rank	5^a^	3.00	15.00	−2.023^d^	.043^∗^
	Positive rank	0^b^	.00	.00		
	Knot	0^c^				
	Total	5				

**Table 2:** Signed-rank sum test results of ATEC total score of children in control group.

		*N*	Rank mean	Rank sum	*Z*	Asymptotic significance (bilateral)
ATEC total score posttest —ATEC total score pretest	Negative rank	3^a^	3.00	9.00	−1.473^d^	.141
	Positive rank	0^b^	1.00	.00		
	Knot	0^c^				
	Total	5				

**Table 3:** Signed-rank sum test results of the scores of each subscale of ATEC in the experimental group.

		*N*	Rank mean	Rank sum	*Z*	Asymptotic significance (bilateral)
ATEC total score posttest —ATEC total score pretest	Negative rank	5^a^	3.00	15.00	−.2.041^d^	.041^∗^
	Positive rank	0^b^	.00	.00		
	Knot	0^c^				
	Total	5				
ATEC total score posttest —ATEC total score pretest	Negative rank	5^a^	3.00	15.00	−.2.023^d^	.043^∗^
	Positive rank	0^b^	.00	.000		
	Knot	0^c^				
	Total	5				

**Table 4:** Signed-rank sum test results of the scores of each subscale of ATEC in children in the control group.

		*N*	Rank mean	Rank sum	*Z*	Asymptotic significance (bilateral)
ATEC total score posttest —ATEC total score pretest	Negative rank	5^a^	2.00	2.00	−.447^d^	.655
	Positive rank	0^b^	1.00	1.00		
	Knot	0^c^				
	Total	5				
ATEC total score posttest —ATEC total score pretest	Negative rank	5^a^	2.50	7.50	−1.000^d^	.317
	Positive rank	0^b^	2.50	2.50		
	Knot	0^c^				
	Total	5				

## Data Availability

No data were used to support this study.
